This article has been retracted.

# Effect of Ghrelin Intervention on the Ras/ERK Pathway in the Regulation of Heart Failure by PTEN

**DOI:** 10.1155/2022/1045681

**Published:** 2022-01-17

**Authors:** Yong Zhao, Quan Sun, Zhenyu Xu, Meixiu Li, Guozhong Tian

**Affiliations:** ^1^Key Laboratory of Microecology-Immune Regulatory Network and Related Diseases, School of Basic Medicine, Jiamusi University, Jiamusi 154007, China; ^2^Department of Anatomy, School of Basic Medicine, Jiamusi University, Jiamusi 154007, China

## Abstract

**Objective:**

To study the possible mechanism of ghrelin in heart failure and how it works.

**Method:**

In vitro results demonstrated that ghrelin alleviates cardiac function and reduces myocardial fibrosis in rats with heart failure. Moreover, ghrelin intervention increased PTEN expression level and reduced ERK, c-jun, and c-Fos expression level; in vivo experiments demonstrated that ghrelin intervention reduces mast memory expression and increases cardiomyocyte surface area, PTEN expression level, ERK, c-jun, c-Fos expression level, and cell surface area, while ERK blockade suppresses mast gene expression and reduces cell surface area.

**Results:**

In vitro experimental results prove that we have successfully constructed a rat model related to heart failure, and ghrelin can alleviate the heart function of heart failure rats and reduce myocardial fibrosis. In addition, ghrelin is closely related to the decrease of the expression levels of ERK, c-jun, and c-Fos, but it can also increase the expression of PTEN in the rat model; in vivo experiments proved that we successfully constructed an in vitro cardiac hypertrophy model, and the intervention of ghrelin would reduce the expression of hypertrophic memory and increase the surface area of cardiomyocytes, increase the expression level of PTEN, and reduce the expression levels of ERK, c-jun, and c-Fos, while the blockade of PTEN will increase the expression of hypertrophy genes and increase the cell surface area, while the blockade of ERK will increase the expression of hypertrophic genes, which in turn will make the cell surface area reducing.

**Conclusion:**

Ghrelin inhibits the phosphorylation and nuclear entry of ERK by activating PTEN, thereby controlling the transcription of hypertrophic genes, improving myocardial hypertrophy, and enhancing cardiac function.

## 1. Introduction

Myocardial dysfunction is an important feature of cardiomyopathy caused by many reasons. Myocardial dysfunction eventually leads to heart failure (HF) [1]. Genetic factors are also a key factor in the occurrence of heart failure. In addition, high blood pressure, diabetes, and obesity can also increase heart pressure and lead to heart failure [2].

In 1999, researchers discovered ghrelin in the stomach of rats for the first time. It can participate in the regulation of various life activities of the human body and play an important role in energy balance and weight maintenance. Ghrelin is a kind of growth hormone releasing peptide, and it is also a ligand affected by growth hormone secretagogue [3, 4]. At present, studies have found that ghrelin can also play a certain role in the treatment of cardiovascular diseases, including regulating sympathetic nerve activity and hypertension, enhancing vascular activity and angiogenesis, inhibiting arrhythmia, reducing heart failure, and inhibiting cardiac remodeling after myocardial infarction [4] . The cardiovascular protective effect of ghrelin may be related to anti-inflammatory, antiapoptosis, inhibition of sympathetic nerve activation, regulation of autophagy, and endothelial dysfunction [5]. However, the relationship between ghrelin and the cardiovascular system has not been elaborated in the relevant literature; so, it is very important to further explore the pharmacology of ghrelin to regulate and treat cardiovascular diseases.

In this article, we have explored the therapeutic effect of ghrelin on myocardial failure and the underlying molecular mechanism through in vivo and in vitro experiments, providing a basis for ghrelin's treatment of myocardial failure.

## 2. Materials and Methods

### 2.1. Establish a Rat Model of Heart Failure

80 SD rats were purchased from the Experimental Animal Center of Harbin Medical University. All 80 rats were female, healthy, and weighing 200-220 g. The rats were fed at the Animal Experiment Center of Jiamusi University at a temperature of 22 ± 2°C and natural light. The rats could eat and drink freely. During the experiment, there were 8 mice in each group. The normal control group (Ctrl group) and the sham group (sham group) did not ligate the left anterior descending coronary artery. The group constructed a rat model of heart failure after myocardial infarction and then ligated the left anterior descending coronary artery. After 4 weeks of culture, the surviving rats were divided into the heart failure model group (HF group, *n* = 27) and ghrelin intervention group (HF + Ghr group, *n* = 27). The rats in the HF + Ghr group were injected with 100 *μ*g/kg ghrelin daily through the tail vein, and the other groups were injected with the same amount of normal saline.

### 2.2. Establish a Model of Cardiomyocyte Hypertrophy

The cardiomyocytes H9C2 were cultured in DMEM medium containing 10% fetal bovine serum FBS, and the culture environment was stable, maintaining a 5% CO_2_ concentration and 37°C room temperature.. Cell growth was observed under an inverted microscope, and conduction was conducted when the cell density reached 80%-90%. H9C2 cells in logarithmic growth phase were selected and randomly divided into 9 groups and cultured in a 12-well plate at 2 × 105 cells/ml for 24 hours: (1) No intervention in the control group; (2) normal cells + ghrelin (3) Ang II group, medium with AngII; (4) Ang II + ghrelin group, medium with AngII and ghrelin; (5) Ang II + PTEN blocking group, medium with AngII and SF1670 (PTEN blocker); (6) AngII + GHRP + PTEN block group, medium with AngII, ghrelin, and SF1670; (7) AngII + ERK block group, medium with AngII and U0126 (ERK blocker); (8) AngII + ghrelin + ERK blocking group, medium plus AngII, ghrelin, and U0126; and (9) AngII + ghrelin + PTEN blocking + ERK blocking group, medium plus AngII, ghrelin, SF1670, and U0126. Among them, the working concentrations of ghrelin, AngII, SF1670, and U0126 are 100 nmol/L, 10umol/L, and 10umol/L, respectively.

### 2.3. Evaluation of Rat Heart Function by Echocardiography

After 4 weeks of intervention in the rats, the rats in each group were subjected to echocardiography, and their cardiac function was evaluated. 50 mg/kg pentobarbital was injected intraperitoneally. After anesthesia, the rat was fixed, and the rat's thoracic hair was removed with a shaving knife. The echocardiogram was monitored on the left side of the rat supine and records the left ventricular end-diastolic diameter (LVEDD), left ventricular end systolic volume (LVESV), left ventricular end systolic diameter (LVESD), left ventricular shortening rate (LVFS), left ventricular end diastolic volume (LVEDV), and left ventricular ejection fraction (LVEF).

### 2.4. Real-Time q-PCR Detection of mRNA Expression

TRIzol (purchased from invitrogen) was used to extract RNA from rat cardiomyocytes, and the concentration of RNA was determined by the nanodrop method. See Table 1 for the sequence of RNA reverse transcription primers.

### 2.5. Western Blot Detection of the Expression of BNP, PTEN, ERK, c-jun, and c-Fos

Myocardial tissue protein collection: collect rat myocardial tissue, add 500 μl cold RIPA buffer, lyse on ice for 30 minutes after the tissue disruptor, 4°C, 3000 g, and centrifuge for 10 min to collect the supernatant. Cardiomyocyte protein collection: after collecting the cells, wash 3 times with 1 ml PBS, 500 g, 3 min, add 50 μl cell lysate containing protease inhibitor and phosphatase inhibitor, lyse on ice for 10 minutes, collect the cells, shake well and then ice bath for 10 repeat 3 times, 4°C, 3000 g, and centrifuge for 10 min to collect the supernatant. BCA method detects protein concentration. Separate equal amounts of protein on 12% SDS-PAGE electrotransfer to nitrocellulose membrane, block with 3% skimmed milk TBST for 2 hours, and incubate with primary antibody (1 : 500) overnight. Wash the cell membrane with TBST and incubate with HRP-conjugated secondary antibody (1 : 200) after 3 washes. When detecting membranes, chemiluminescence (ECL) western blot detection methods are used.

### 2.6. Masson Staining

The rat heart tissue was fixed with 4% paraformaldehyde, and the PFA was washed away and then processed by a series of steps such as dehydration, wax immersion, embedding, and sectioning. Then, the paraffin sections were deparaffinized with water, and the nuclei were stained with hematoxylin and ponceau and then stained with phosphomolybdic acid, aniline blue, differentiation, dehydration, sealing, drying, and a series of operations to produce The specimen is placed under a microscope for observation.

### 2.7. Immunohistochemical Staining

1.7.1 Bake the paraffin sections made in the first step of the above steps at 60°C for 1 hour, wash 3 times in distilled water, repair in a microwave oven, then cool to room temperature, and wash 3 times with PBS (5 minutes each time)

1.7.2 The sections are sealed in 5% BSA and room temperature for 20 minutes. Drop the primary antibody in 1 h and wash with PBS 3 times, 3 min each time; drop the secondary antibody in 15-30 min and wash 3 times with PBS, 3 min each time. Add SABC dropwise in 30 min and wash 3 times with PBS, 5 min each time. Finally, add color reagent dropwise, mixing

1.7.3 After adding DAB color reagent to react for 5 minutes, rinse with tap water and distilled water, respectively, then counterstain with hematoxylin for 2 minutes, and rinse off excess hematoxylin dye with tap water

1.7.4 Dehydrate the sections and fix them on a glass slide with glue and observe under a microscope

### 2.8. Immunofluorescence Staining

Collect the cells in the cell culture medium, rinse with PBS solution, add 2 ml 4% paraformaldehyde, and incubate at room temperature for 20 minutes; rinse 3 times with 2 ml PBS, 5 minutes each time; permeabilize with 2 ml PBS-T solution at 4°C. Incubate the cells for 10 minutes; rinse the PBST solution from the cells with PBS for 5 minutes; block nonspecific interaction with PBS-B solution at 37°C; add the primary antibody solution after 30 minutes and incubate overnight at 4°C; wash with PBS to remove the primary antibody solution; add the secondary antibody solution and incubate at room temperature for 1 hour; then, wash with PBS 3 times and observe.

### 2.9. Statistical Analysis

Analyze the experimental data with SPSS 22.1, and the results are expressed as mean ± standard deviation. The independent sample *t*-test was used to compare the two groups, and the *F* test was used to compare multiple groups. *P* < 0.05 indicates that the data difference between the groups is statistically significant.

## 3. Results

### 3.1. Ghrelin Effectively Improves Heart Function in Rat Models of Heart Failure

Table 2 indicates cardiac function indexes of the rat heart failure model after different treatments. The experimental data showed that LVEDD, LVEF, LVESD, LVESV, LVEDV, and LVFS in the HF group were increased compared with the Ctrl group and the sham group (*P* < 0.05); that is, the rat heart failure model is effective and feasible, which can also be seen from the echocardiogram results in Figure 1. Although the heart function of the HF + Ghr group treated with ghrelin was worse than that of the Ctrl group and the sham group, it was still improved compared to the HF myocardial failure model. We detected the heart function of the rat model by echocardiography in the 4th week, and we can see that ghrelin helps to improve the heart function of the rat heart failure model.

Heart function in the HF + Ghr group, although inferior to the Ctrl and Sham groups, was still improved compared to the HF myocardial failure model.

### 3.2. Ghrelin Reduces Myocardial Fibrosis in a Rat Model of Heart Failure

After detecting the improvement of ghrelin on the cardiac function of the rat heart failure model by echocardiography, we further observed the effect of ghrelin on myocardial tissue fibrosis at the tissue level. It can be seen from Figure 2 that the myocardial fiber structure of the rats in the Ctrl and sham groups can be clearly observed under an optical microscope, while the myocardial cells of the HF group have hypertrophy, thickened myocardial fibers, and disordered arrangement of myocardial cells. There are clear horizontal and vertical lines, and there are obvious differences between normal cells. In addition, the cardiomyocytes of the HF group have a large amount of inflammatory cell infiltration. The clarity of myocardial fibers in rats was in the order of Ctrl group, HF + Ghr group, and HF group. The number of hypertrophic cardiomyocytes and the number of inflammatory cells in the HF + Ghr group were improved. It can be seen from this that ghrelin can not only improve the myocardial function of rats but also reduce the degree of myocardial tissue fibrosis in rats.

The myocardial fibers in rats in Ctrl and sham had clear fiber structure, clear transverse, and longitudinal lines and normal cell morphology.

### 3.3. Ghrelin Relieves Rat Heart Function by Upregulating the Expression of PTEN Protein and Reducing the Phosphorylation of Ras and ERK

Ghrelin can alleviate the heart function of the rat heart failure model, reduce myocardial fibrosis, and improve myocardial cell hypertrophy. In order to study the role of ghrelin in the pathogenesis of heart failure, we obtained the myocardial tissue of a rat model, and extracted the protein in the tissue, and with the help of a series of methods to detect the possible molecular mechanism of ghrelin from the level of protein and RNA, such as immunohistochemistry, Western blot, real-time quantitative PCR, and other methods. Firstly, p-ERK is expressed in the cytoplasm and nucleus of tissue cells. As shown in Figure 3, the expression level of p-ERK was the highest in the HF group, which was significantly better than the Ctrl group and the sham group, while the expression level was the lowest in the ghrelin group, and it was almost not expressed in rats with early-onset heart failure. The expressions of p-PTEN and p-ERK were opposite, not only recovered in the ghrelin group but even higher in expression than the Ctrl group and the sham group. In view of the abnormal expression of p-PTEN and p-ERK in myocardial tissue, we extracted protein and RNA from myocardial tissue and performed semiquantitative analysis. Consistent with the results observed in myocardial tissues, compared with the Ctrl group and the sham group, ERK was expressed at a higher level in the cardiomyocytes of heart failure rats, and ghrelin could downregulate the expression of ERK in heart failure rats. The expression of p-PTEN is just the opposite, and this response is consistent with the response of the heart failure marker BNP.

In early studies, it has been suggested that ghrelin can improve myocardial function through the PTEN/PI3K/Akt pathway, but it has not been reported that ERK is also involved in the process of ghrelin in improving heart failure. As we all know, ERK participates in the Ras signaling pathway, and the phosphorylation of ERK is essential for cell transcription. Therefore, here we further use experiments to prove the expression of nuclear transcription factors at the protein and RNA levels in Figures 4 and 5. As we guessed, the expression levels of nuclear transcription factors c-Fos and c-jun in the cardiomyocytes of rats with heart failure were significantly upregulated. This upregulation may promote the expression of hypertrophy-related genes in cardiomyocytes, and treatment with ghrelin can reverse c-jun and c -Fos upregulation.

### 3.4. Ghrelin Reduced the Expression of Hypertrophic Genes (ANP, *β*-MHC) in Cardiac Mast Cell Model

After proving the effect and potential mechanism of ghrelin on the heart function of rats with heart failure in an in vivo model of heart failure rats, we constructed a cardiac mast cell model. As we mentioned above, ghrelin may inhibit the phosphorylation of ERK, thereby inhibiting the expression of hypertrophic genes in the nucleus of cardiomyocytes. In order to verify our conjecture, we first detected the expression of the hypertrophic genes ANP and *β*-MHC in the cardiac mast cell model. In Figure 6, the research data represents that the treatment of ghrelin can reduce the expression of the hypertrophic genes ANP and *β*-MHC. In addition, we also used immunofluorescence staining to capture the cell morphology of the cardiac mast cell model and obtained semiquantitative results. From Figure 7, we can see that ghrelin can effectively reduce the cell surface area of the cardiac mast cell model. In addition, in Figure 8, we also tested the heart failure marker BNP in the cell model, and the results are consistent with the in vivo model.

### 3.5. Ghrelin Upregulated the Expression of PTEN in the Cardiac Mast Cell Model and Downregulated the Phosphorylation of ERK

After evaluating the in vitro cardiac mast cell model and the effect of ghrelin, we further verified the previous conjecture in the in vitro model. Similarly, we also observed in the in vitro cardiac mast cell model that p-ERK, pc-Fos, and c-jun are elevated in the cardiac mast cell model, and ghrelin treatment reduces the expression of these molecules, while the expression of PTEN significantly increased after ghrelin treatment.

### 3.6. PTEN Blocker SF1670 or ERK Blocker U0126 Reversed the Alleviating Effect of Ghrelin on Myocardial Hypertrophy

From the above results, we have already observed the response of PTEN/ERK expression after ghrelin treatment, but is this response caused by ghrelin treatment? In order to further prove that ghrelin does indeed inhibit the Ras/ERK signaling pathway by activating PTEN, thereby inhibiting the transcription of myocardial hypertrophy-related genes, thereby improving cardiac function, we added PTEN blocker SF1670 and ERK blocker U0126 to the in vitro cardiomyocyte mast cell model and detected the expression of hypertrophic genes ANP, *β*-MHC, and PTEN, ERK, c-jun, and c-Fos in cardiomyocytes. Simultaneously detect the morphology and cell surface area of cardiomyocytes.

As can be seen from the results, as shown in Figure 6, the blockade of PTEN does not reduce the expression of hypertrophic genes caused by Ang II, but also reduces the expression of hypertrophic genes after ghrelin treatment, indicating that the blockade of PTEN leads to ERK dephosphorylation. When it is inhibited, the process of ERK entering the nucleus is enhanced, and the expression of hypertrophic genes is upregulated. This cascade reaction will not be blocked by ghrelin, because ghrelin plays a role upstream of PTEN. In contrast, ERK phosphorylation blockers reduce the expression of hypertrophic genes caused by Ang II, and the addition of ghrelin will enhance this downregulation effect; it means that blocking ERK phosphorylation is to inhibit ERK from entering the nucleus, making it difficult to upregulate the expression of hypertrophic genes. As shown in Figure 9 and Table 3, the upregulation or downregulation of this hypertrophy gene is consistent with the change in the relative surface area of cardiomyocytes.

Similarly, the blocking effect of PTEN affects the expression of PTEN in cardiomyocytes, but also enhances the expression of c-Fos, ERK and c-jun, while the effect of ERK is the opposite of PTEN.

## 4. Discussion

Heart failure is due to insufficient blood perfusion in the arterial system caused by the diastolic or diastolic dysfunction of the heart, which causes cardiac circulatory disorders [2]. The cause of myocardial failure is complex, as long as it can cause changes in myocardial damage, and it will lead to myocardial failure, such as myocardial infarction, arrhythmia, inflammation, cardiomyopathy, and myocardial failure caused by some drugs, such as digitalis [6, 7]. The electrocardiogram of patients with acute myocardial failure is mainly manifested as left ventricular enlargement and galloping rate in the early and middle diastole. Clinical detection and diagnosis mainly rely on electrocardiogram and echocardiography, and B-type natriuretic peptide (BNP) is also an important marker of heart failure [8, 9]. In clinical treatment of acute myocardial failure, most of them choose to use vascular activating drugs, while the treatment of chronic myocardial failure is mainly based on long-acting repair neuroendocrine inhibitors [9]. Current research is also actively developing other strategies for the treatment of myocardial failure, such as promoting the endogenous repair of the heart by regulating the cell biological processes in the proliferation and regeneration of myocardial cells.

In our study, the left coronary artery of SD male rats was ligated anteriorly to simulate the symptoms of left coronary artery stenosis or occlusion, leading to myocardial ischemia and infarction, and ultimately leading to heart failure due to decreased myocardial contractility. Using echocardiography to detect the recovery of rat heart function, Masson staining to observe myocardial fibrosis, it was found that ghrelin can effectively improve the function of rat cardiomyocytes. Myocardial fibrosis is the main cause of heart remodeling and an important factor leading to heart failure and death. Ghrelin can not only improve the heart function of the rat heart failure model, but also improve the fibrosis of the rat myocardial tissue, which is very important for alleviating the long-term heart pressure of patients with chronic myocardial failure. This result is not surprising, because ghrelin has been shown to treat cardiovascular diseases, including reducing heart failure. But here, we have carried out a series of explorations on the mechanism of ghrelin in the treatment of heart failure. Different from AKT/PI3K and Nrf2/NADPH/ROS [4, 10] that have been reported, our study found that the way ghrelin works is more complicated, involving not only PTEN/AKT/PI3K but also ERK signaling pathways. This kind of complex network communication is more conducive to the stable regulation of ghrelin.

The PI3K-Akt/PKB pathway is an important mechanism of heart failure, and the signal transduction family of phosphoinositide 3-kinase (PI3K) and its downstream target serine/threonine kinase protein kinase B (Akt/PKB) play an important role. PTEN blockade does not reduce the expression of mast genes caused by Ang II, but also after ghrelin treatment, indicating that PTEN blockade causes inhibition of dephosphate of ERK, enhanced nucleation process, and elevated mast gene expression. This cascade is not blocked by ghrelin because it functions upstream of PTEN. A number of studies and documents have proved that this pathway is the center of the signal transduction pathway and plays an important role in regulating inflammation, apoptosis, and cell activation [11]. At the same time, PI3K and Akt are also the key to promote the survival of cardiomyocytes and give full play to the function of cardiomyocytes [12]. The blocking of activation of this signaling pathway mainly relies on the negative regulation of chromosome 10 phosphatase and tensin homolog (PTEN) deletion, which dephosphorylates PIP3 to PIP2 [13, 14]. In addition, there are some signal transduction pathways that also play a key role in cell proliferation, transformation, and apoptosis, such as the extracellular signal-regulated kinase (ERK1/2) pathway [15]. The protective effect of ERK phosphorylation in the heart has also been reported, but whether ghrelin can trigger this protective effect is unknown.

It must be emphasized that PTEN, as a dual-specific phosphatase, can dephosphorylate lipids and proteins on serine, threonine, and tyrosine residues in many tissues including heart and cardiomyocytes and widely expressed in cells [13]. In recent years, with the deepening of research on PTEN, more and more biological functions have been recognized, including embryonic development, tumorigenesis, and heart growth. In 2002, Crackower found that PTEN can reduce the contractility of cardiomyocytes and increase the possibility of myocardial hypertrophy when inactivated [14].

The PI3K/Akt and ERK signaling pathways are important central signal transduction pathways. Their mechanism of action is to improve the survival rate of cardiomyocytes and maintain the normal physiological functions of the myocardium by regulating the levels of cell proliferation and apoptosis and regulating protein synthesis and metabolic integration [12, 15]. In this study, we demonstrated the upregulation of ghrelin on PTEN. Upregulation of PTEN can not only inhibit the activation of PI3K/Akt but also inhibit the phosphorylation of ERK, thereby inhibiting the activation of transcriptional regulators such as AP-1 in the nucleus. The end result is that the activation of genes for cardiomyocyte hypertrophy is inhibited. Ghrelin may inhibit the phosphorylation of ERK and the transmission of downstream signals by upregulating PTEN, but there is no more evidence to prove the way PTEN inhibits ERK phosphorylation, and whether it affects downstream molecules c-jun and c-Fos by inhibiting nuclear localization. What effect does this effect have on the apoptosis or proliferation of cardiomyocytes? The research results and experimental data of this experiment have far-reaching significance for confirming that ghrelin can effectively treat heart failure and are also the main key points of future experimental research. However, the current evidence supports our hypothesis that the upregulated expression of PTEN may dephosphorylate ERK2, making ERKs unable to effectively form homodimers. We all know that homodimers of ERKs are necessary for the transfer of ERK from the cytoplasm to the nucleus. Once ERKs homodimers fail to form, nuclear transcription factors are not activated, and genes related to cardiomyocyte hypertrophy cannot initiate transcription.

## Figures and Tables

**Figure 1:** The echocardiogram of each group of rat models.

**Figure 2:** Masson staining pathological imaging results of myocardial tissue of rats in each group (×400).

**Figure 3:** ERK and PTEN immunohistochemical staining results of cardiomyocytes in different groups of rat models.

**Figure 4:** The results of Western blot extraction of cardiomyocyte protein in different groups of rat models. Note: ^∗^compared with the Ctrl group, *P* < 0.05; &compared with the HF group, *P* < 0.05; #compared with the HF + Ghr group, *P* < 0.05.

**Figure 5:** Real-time quantitative PCR measurement results of rat model cardiomyocyte RNA in different groups.

**Figure 6:** Real-time quantitative PCR detection of RNA expression of hypertrophic genes (ANP, *β*-MHC) in the cardiac mast cell model.

**Figure 7:** Western blot detection of the expression of ERK and other molecules in cardiac mast cells. Note: groups 1-9 are the control group, AngII+ ghrelin, AngII group, AngII+ PTEN blocking group, AngII+ ghrelin+ PTEN blocking group, AngII+ ghrelin+ ERK blocking group, AngII+ ERK blocking group, AngII+ ghrelin + PTEN blocking + ERK blocking group, and ghrelin group.

**Figure 8:** Real-time quantitative PCR detects the expression levels of ERK and other molecules in cardiac mast cells. Note: ^∗^compared with the Ctrl group, *P* < 0.05; ∆compared with the AngII+ghrelin group, *P* < 0.05; ∆compared with the AngII+SF1670 group, *P* > 0.05; #compared with the AngII group, *P* < 0.05.

**Figure 9:** Cellular immunofluorescence results of myocardial mast cell model.

**Table 1:** Primer sequence of each gene.

Gene	Primer sequence(5′⟶3′)
BNP	Upstream: GGACAACCTCCCTAGACCCT
	Downstream: GCATCTGGCTTTCGTCTTGG
PTEN	Upstream: CAATATCCTTTTTGCCATAACC
	Downstream: TGCCCCGATGTAAATATGC
erk1/2	Upstream: TACACCAACCTCTCGTACATCG
	Downstream: CATGTCTGAAGCGCAGTAAGATT
c-Fos	Upstream: GGTCATCGGGGATCTTGC
	Downstream: GGGCTCTGTCAA
c-jun	Upstream: GATGGAAACGACCTTCTACG
	Downstream: GTTGAAGTTGCTGAGGTTG

**Table 2:** Comparison of LVEDD, LVESD, LVEDV, LVESV, LVEF, and LVFS in each group (±*s*).

Groups	LVEDD	LVESD	LVEDV	LVESV	LVEF (%)	LVFS (%)
Ctrl	6.69 ± 0.19	2.92 ± 0.13	218.38 ± 14.28	27.98 ± 3.21	87.37 ± 0.62	56.6 ± 0.72
Sham	6.65 ± 0.02	2.74 ± 0.10	222.14 ± 1.58	28.34 ± 2.52	87.39 ± 1.09	58.88 ± 1.40
HF	9.50 ± 0.14^∗^^#^	7.77 ± 0.78^∗^^#^	504.75 ± 16.37^∗^^#^	281.39 ± 6.10^∗^^#^	44.84 ± 0.64^∗^^#^	23.09 ± 0.41^∗^^#^
HF + Ghr	8.25 ± 0.14^∗^^#^	5.95 ± 0.12^∗^^#@^	410.36 ± 14.67^∗^^#^	177.01 ± 8.20^#^^∗^^@^	56.88 ± 0.41^∗^^#@^	31.19 ± 0.25^∗^^#@^

Note: compared with the Ctrl group, ^∗^*P* < 0.05; compared with the HF group, ^@^*P* < 0.05; compared with the sham group, ^#^*P* < 0.05.

**Table 3:** Comparison of cardiomyocyte surface area in each group ($\bar{x}\pm s$).

Groups	Cell surface area (*μ*m^2^)
Ctrl	103.57 ± 13.53
Ghrelin	104.09 ± 11.80^∆^
AngII	397.62 ± 28.11^∗^
AngII+ ghrelin	147.23 ± 15.62^#^
AngII+ SF1670	409.33 ± 23.35^∗^
AngII+ ghrelin + SF1670	389.02 ± 21.87^∗^
AngII+ U0126	132.56 ± 10.21^#^
AngII+ ghrelin + U0126	109.42 ± 9.55^#^

Note: ∗compared with the Ctrl group, *P* < 0.05; #compared with the AngII group, *P* < 0.05; ∆ compared with the control group, *P* > 0.05.

## Data Availability

The data used to support the findings of this study are included within the article.
